# Artificial and bioartificial liver support systems for acute and acute-on-chronic hepatic failure: A meta-analysis and meta-regression

**DOI:** 10.3892/etm.2013.1241

**Published:** 2013-07-31

**Authors:** ZHEN ZHENG, XU LI, ZHILIANG LI, XIAOCHUN MA

**Affiliations:** Department of Intensive Care Unit, The First Hospital, China Medical University, Heping, Shenyang, Liaoning 110001, P.R. China

**Keywords:** liver support systems, hepatic failure, meta-analysis, meta-regression

## Abstract

Artificial and bioartificial liver support systems (LSSs) appear to be safe and effective in the treatment of acute and acute-on-chronic hepatic failure (AHF and AOCHF); however, individually published studies and previous meta-analyses have revealed inconclusive results. The aim of the present meta-analysis was to derive a more precise estimation of the benefits and disadvantages of artificial and bioartificial LSSs for patients with AHF and AOCHF. A literature search was conducted in the PubMed, Embase, Web of Science and Chinese Biomedical (CBM) databases for publications prior to March 1, 2013. Crude relative risks (RRs) or standardized mean differences (SMDs) with 95% confidence intervals (95% CI) were calculated using either the fixed effects or random effects models. Nineteen randomized controlled trials (RCTs) were included, which comprised a total of 566 patients with AHF and 371 patients with AOCHF. The meta-analysis showed that artificial LSS therapy significantly reduced mortality in patients with AOCHF; however, it had no apparent effect on total mortality in patients with AHF. The results also indicated that the use of bioartificial LSSs was correlated with decreased mortality in patients with AHF. A significant reduction in the bridging to liver transplantation was observed in patients with AOCHF following artificial LSS therapy; however, similar results were not observed in patients with AHF. Patients with AHF and those with AOCHF showed significant reductions in total bilirubin levels following artificial LSS therapy. There were no significantly increased risks of hepatic encephalopathy or bleeding in either the patients with AHF or AOCHF following artificial or bioartificial LSS therapies. Univariate and multivariate meta-regression analyses confirmed that none of the factors explained the heterogeneity. The present meta-analysis indicated that artificial LSSs reduce mortality in patients with AOCHF, while the use of bioartificial LSSs was correlated with reduced mortality in patients with AHF.

## Introduction

Acute hepatic failure (AHF) is a severe liver injury accompanied by hepatic encephalopathy, which leads to multi-organ failure with an extremely high mortality rate (1). Acute-on-chronic hepatic failure (AOCHF) has been defined as an acute deterioration of liver function in chronic liver disease that ultimately leads to multi-organ failure within 4–6 weeks, with a mortality rate of 53% (2). Liver transplantation has long been recognized as the most effective therapy in the treatment of AHF and AOCHF (3). However, this therapeutic strategy is limited by the insufficient organ resources and a significantly elevated demand for liver transplantation. Therefore, extracorporeal liver support systems (LSSs), as an alternative source for liver transplantation, have attracted increased focus over the last four decades (4).

Artificial LSSs were originally developed in Germany and were designed to remove toxic substances from the blood that would normally be filtered out by a functioning liver (5). Artificial LSSs transport a patient’s blood through a filter where it is mixed with albumin. The toxins and metabolic waste from the blood that are mixed with the albumin molecules are then carried out of the blood (6). Bioartificial LSSs, which are essentially bioreactors, utilize either human hepatocytes or porcine liver cells to process oxygenated blood plasma, which is subsequently separated from the other blood constituents (7). The aim of artificial and bioartificial LSSs is to temporarily replace liver functions until a transplant is available (8). It has been demonstrated that artificial and bioartificial LSSs are important in the improvement of jaundice, the amelioration of hemodynamic instability, the reduction of portal hypertension, the lowering of intracranial pressure and the reduction in short-term mortality in patients with AHF and AOCHF (9). Moreover, in cases of hepatic encephalopathy, patients have shown marked reductions in ammonia levels, clearance of aromatic amino acids and improvements in systemic hemodynamics, which may partially explain the potential benefits of artificial and bioartificial LSSs in improving hepatic encephalopathy in patients with hepatic failure (10). Previous meta-analyses have demonstrated that artificial and bioartificial LSSs may lead to significant improvements in total bilirubin levels, hepatic encephalopathy, the incidence of bleeding and bridging to transplantation (11–13). However, the results remain debatable with regard to whether artificial and bioartificial LSSs are able to improve survival in patients with AHF or AOCHF. These inconsistent results may be due to the limited number of studies and relatively small number of patients suitable for study in the previous meta-analyses. Therefore, in the present study, an updated meta-analysis was performed on all the eligible literature to evaluate the benefits and harmful effects of artificial and bioartificial LSSs in patients with AHF and AOCHF.

## Materials and methods

### Literary search

Relevant papers published prior to March 1, 2013 were identified through a search of the PubMed, Embase, Web of Science and Chinese Biomedical (CBM) databases using the following terms: (‘liver support system’ or ‘liver, artificial’ or ‘artificial liver’ or ‘bioartificial liver’ or ‘extracorporeal liver’) and (‘hepatic failure’ or ‘liver failure’ or ‘liver failure, acute’ or ‘liver failure, acute’ or ‘end stage liver disease’ or ‘liver failure, chronic’). The references used in eligible articles or textbooks were also reviewed to examine other potential sources. Disagreements were resolved through discussions between the authors.

### Inclusion and exclusion criteria

Studies included in the meta-analysis had to meet the following criteria: i) randomized controlled trials (RCTs) focused on the effects of artificial and bioartificial LSSs in patients with AHF and AOCHF; ii) study populations included patients with AHF and AOCHF; iii) interventions (treatment groups) included artificial and bioartificial LSSs, while the comparison intervention (control group) used standard medical therapy, including electrolyte substitution, fluid substitution, antacid therapy, coagulation therapy and N-acetylcysteine; and iv) published data on the clinical outcomes must be sufficient. The exclusion criteria were as follows: i) not an RCT on the effects of artificial and bioartificial LSSs in patients with AHF and AOCHF; ii) duplicates of previous publications; iii) based on incomplete data; and iv) meta-analyses, letters, reviews and editorial articles. If more than one study by the same author using the same case series was published, either the study with the largest sample size or the most recently published study was included.

### Data extraction

Data from the published studies were extracted independently by two authors into a standardized form. For each study, the following characteristics and numbers were collected: first author, year of publication, country, language, study design, numbers of subjects, subtype of hepatic failure, inclusion criteria for subjects, type of liver support system, duration of follow-up, outcomes and methodological quality. In cases of conflicting evaluations, disagreements were resolved through discussions between the authors.

### Study outcome

All outcomes were assessed subsequent to the maximum follow-up. The following outcome data were extracted from the studies: i) mortality; ii) bridging to liver transplantation; iii) total bilirubin levels; iv) hepatic encephalopathy; and v) incidence of bleeding.

### Methodological quality assessment

This meta-analysis was performed according to recommendations from the Preferred Reporting Items for Systematic Reviews and Meta-analyses (PRISMA) statement (14). Two authors independently assessed the quality of the papers according to the Consolidated Standards of Reporting Trials (CONSORT) criteria (15). A point was awarded for each criterion met. The mean CONSORT score was calculated for each trial. Disagreements were resolved through discussions between the authors.

### Statistical analysis

Crude relative risks (RRs) or standardized mean differences (SMDs) with 95% confidence intervals (95% CI) were calculated for dichotomous outcomes and continuous outcomes, respectively. The statistical significance of the pooled value was examined using the Z-test. Interstudy variations and heterogeneities were estimated using Cochran’s Q-statistic with P<0.05 as a cutoff for statistically significant heterogeneity (16). The effects of heterogeneity were also quantified using the I^2^ test, which ranges from 0 to 100% and represents the proportion of interstudy variability that may be contributed to heterogeneity rather than by chance (17). When a significant Q-test (P<0.05) or I^2^ >50% indicated that heterogeneity existed among the studies, the random effects model (DerSimonian-Laird method) was conducted for meta-analysis; otherwise, the fixed effects model (Mantel-Haenszel method) was used. To explore sources of heterogeneity, univariate and multivariate regression analyses were also performed (18). A sensitivity test was performed by omitting each study randomly and assessing the stability of the results. Begg’s funnel plot and Egger’s linear regression test were used to evaluate the publication bias (19). All P-values were two-sided and P<0.05 was considered to indicate a statistically significant difference. All analyses were calculated using STATA statistical software version 12.0 (Stata Corp., College Station, TX, USA).

## Results

### Characteristics of included studies

In accordance with the inclusion criteria, 19 RCTs (20–38) were assessed in this meta-analysis and 113 studies were excluded. The publication years of the included studies ranged from 1973 to 2012. A flow chart of the study selection process is shown in Fig. 1. A total of 937 patients with hepatic failure were involved in this meta-analysis, including 566 patients with AHF and 371 patients with AOCHF. With regard to the therapeutic strategy in the treatment group, 16 studies adopted artificial LSSs while the remaining studies adopted bioartificial LSSs. The control groups received standard medical therapy aimed at preventing the complications associated with severe liver failure. The characteristics and methodological quality of the included studies are summarized in Table I.

### Mortality

Among the 19 included studies, 16 described data on the effects of artificial LSSs on mortality in patients with AHF and AOCHF, while only three studies referred to the effects of bioartificial LSSs on mortality. Meta-analysis showed that artificial LSS therapy significantly reduced mortality in patients with AOCHF (RR= 0.80, 95% CI= 0.66–0.96, P= 0.018). The results also showed that the use of bioartificial LSSs was correlated with decreased mortality in patients with AHF (RR=0.69, 95% CI=0.50–0.94, P=0.018). However, it was observed that artificial LSSs had no apparent effect on total mortality in patients with AHF (RR=0.87, 95% CI=0.71–1.07, P=0.187; Fig. 2).

### Bridging to liver transplantation

Five of the 19 studies described data on the bridging to liver transplantation with artificial LSS therapy. Our meta-analysis demonstrated significant reductions in the bridging to liver transplantation in patients with AOCHF following artificial LSS therapy (RR= 0.66, 95% CI= 0.49–0.90, P= 0.009). However, artificial LSSs had no significant effect on the bridging to liver transplantation in patients with AHF (RR= 0.65, 95% CI= 0.37–1.14, P=0.131; Fig. 3).

### Total bilirubin levels

Seven trials presented data on total bilirubin levels following artificial LSS therapy. Patients with AHF and those with AOCHF were revealed to have significant reductions in total bilirubin levels following artificial LSS therapy (RR= 0.74, 95% CI= 0.48–1.13, P= 0.357; RR=0.60, 95% CI=0.32–1.09, P=0.357, respectively; Fig. 4).

### Hepatic encephalopathy

Nine trials described improvements in hepatic encephalopathy. Patients with AHF and those with AOCHF had no significantly increased risk of hepatic encephalopathy following artificial LSS therapy (RR= 0.76, 95% CI= 0.49–1.16, P= 0.202; RR= 0.64, 95% CI= 0.36–1.15, P= 0.137, respectively). There was also no increased risk of hepatic encephalopathy in patients with AHF following bioartificial LSS therapy (RR= 0.43, 95% CI= 0.14–1.28, P= 0.128).

### Incidence of bleeding

Thirteen trials described the incidence of bleeding. No statistically significant increase in the incidence of bleeding was observed in patients with AHF or AOCHF following artificial LSS therapy (RR=0.97, 95% CI= 0.15–6.19, P= 0.973; RR=1.20, 95% CI= 0.87–1.64, P=0.270, respectively).

### Meta-regression and sensitivity analyses

Univariate and multivariate meta-regression analyses were used to explore possible sources of heterogeneity among the studies (Table II). The results showed that none of the factors explained the heterogeneity (all P>0.05). Sensitivity analysis was performed to assess the stability of the conclusions on the pooled RR of mortality by omitting individual studies. The sensitivity analysis results suggested that no individual study significantly affected the pooled values of the clinical events (Fig. 5), indicating that the results of the meta-analysis were statistically robust.

### Publication bias evaluation

Begg’s funnel plot and Egger’s linear regression test were performed to assess the publication bias of the included studies. The shapes of the funnel plots of mortality did not reveal any evidence of obvious asymmetry (Fig. 6). Egger’s test also displayed no significant statistical evidence of publication bias with regard to mortality (t=−1.02, P= 0.327).

## Discussion

Previous meta-analyses (11–13) have attempted to evaluate the effects of artificial and bioartificial LSSs on the clinical outcomes in patients with AHF and AOCHF; however, the results were inconclusive due to small sample sizes, different study designs, methodological limitations and a wide variety of observed outcome measures. In the meta-analysis by Kjaergard *et al* in 2003 (12), it was revealed that artificial LSSs reduced mortality in patients with AOCHF, while neither artificial nor bioartificial LSSs appeared to affect mortality in patients with AHF. Results from another meta-analysis by Liu *et al* (11) also indicated that artificial LSSs reduced mortality in patients with AOCHF; however, there appeared to be no correlation between the use of artificial or bioartificial LSSs and reductions in mortality in patients with AHF (11). By contrast, in the meta-analysis performed by Stutchfield *et al* (13) in 2011, it was demonstrated that artificial and bioartificial LSSs appeared to improve survival in patients with AHF, although not in patients with AOCHF (13). Therefore, it was imperative to conduct a more systematic and comprehensive meta-analysis to reassess the effects of artificial and bioartificial LSSs on the clinical outcomes of patients with different types of hepatic failure.

In the present study, compared with previous meta-analyses, more stringent inclusion criteria were used (only RCTs were evaluated), more studies were included (19 versus 12 in the analyses by Kjaergard *et al* and Liu *et al*, respectively, and eight in the analysis by Stutchfield *et al*), more patients were assessed (566 with AHF and 371 with AOCHF) and a wider range of eligible articles were analyzed (from 1973 to 2012 compared with from 1973 to 2002 in the study by Kjaergard *et al*, from 1973 to 2001 in the study by Liu *et al* and from 1996 to 2007 in the study by Stutchfield *et al*). The present meta-analysis also evaluated more clinically relevant endpoints (mortality, bridging to transplantation, total bilirubin level, hepatic encephalopathy and bleeding) with greater inferential power. When all available studies were pooled into the present meta-analysis, the results showed that artificial LSS therapy significantly reduced mortality in patients with AOCHF; however, it had no apparent effect on total mortality in patients with AHF. The findings from this meta-analysis were consistent with the previous studies conducted by Kjaergard *et al* (12) and Liu *et al* (11), suggesting that no survival benefits may be derived from artificial LSS therapy for patients with AHF. However, in contrast to the previous meta-analyses, it was observed in the present meta-analysis that the use of bioartificial LSS therapy was correlated with decreased mortality in patients with AHF. Moreover, the current meta-analysis results revealed that there was a significant reduction in the bridging to liver transplantation in patients with AOCHF following artificial LSS therapy, although similar results were not observed in patients with AHF. Significant reductions were observed in total bilirubin levels in the patients with AHF and with AOCHF following artificial LSS therapy, which was consistent with the previous study by Liu *et al* (11). This indicated that an effective clearance of albumin-bound substances was performed in the liver support device (11). There was no significantly increased risk of hepatic encephalopathy in either the patients with AHF or AOCHF following artificial and bioartificial LSS therapies.

Over the past decade, a number of studies have indicated that the use of LSSs may be correlated with several potentially life-threatening adverse effects, including bleeding, infection, coagulopathy and an increase in intracranial pressure, with the most frequently observed adverse effect being bleeding (39,40). However, the result of the present analysis did not reveal any significant increase in the incidence of bleeding in either the patients with AHF or AOCHF following artificial or bioartificial LSS therapy, which was inconsistent with the previous study by Liu *et al* (11). However, in the largest trial of LSSs in patients with AOCHF, published in 2012, there was no difference in the incidence of bleeding between the use of LSSs and standard medical therapy. Despite this, all of the patients in the studies suffered from severe liver disease, so it may be difficult for physicians to conclude whether the LSS therapies or the underlying severe liver disease caused the bleeding. Therefore, additional adequately powered studies addressing these issues in larger populations are required to provide more definitive conclusions.

Similar to other meta-analyses, the present study showed certain limitations, such as a lack of adequate double-blinding procedures. Adequate double-blinding procedures for patients and caregivers were impossible due to the nature of the support systems; this may have increased the risk of false-positive conclusions from the outcomes. In addition, the heterogeneity of the trials included follow-up periods of variable durations and a diverse patient population, with regard to the severity and etiology of the liver failure, which precluded definitive conclusions. Despite these limitations, however, the present meta-analysis also demonstrated several strengths, such as including the largest number of patients with hepatic failure treated with LSSs to date. Moreover, the results were relatively consistent with those observed in the largest study to date and the consistency of the results was maintained in almost each subgroup analysis.

In conclusion, the present updated meta-analysis demonstrated that artificial LSS therapy appeared to reduce mortality in patients with AOCHF, while the use of bioartificial LSS therapy was correlated with decreased mortality in patients with AHF. Artificial LSS therapy also appeared to reduce the bridging to transplantation and levels of total bilirubin; however it did not appear to increase the risks of hepatic encephalopathy and bleeding. Considering the limitations mentioned previously, further adequately powered studies are essential to extend this investigation before any support systems are able to be recommended for routine use.

## Figures and Tables

**Figure 1.** Flow chart of literature search and study selection.

**Figure 2.** Forrest plot on the effects of artificial and bioartificial liver support systems on mortality in patients with acute and acute-on-chronic hepatic failure (AHF and AOCHF). RR, relative risk; CI, confidence intervals.

**Figure 3.** Forrest plot on the effects of artificial liver support systems on bridging to liver transplantation in patients with acute and acute-on-chronic hepatic failure (AHF and AOCHF). RR, relative risk; CI, confidence intervals.

**Figure 4.** Forrest plot on the effects of artificial liver support systems on total bilirubin levels in patients with acute and acute-on-chronic hepatic failure. (AHF and AOCHF). RR, relative risk; CI, confidence intervals.

**Figure 5.** Sensitivity analysis of the summary relative risk coefficients on the effects of artificial liver support systems on mortality. Results were computed by omitting each study in turn. Meta-analysis random-effects estimates (exponential form) were used. The two ends of the dotted lines represent the 95% confidence intervals (CI).

**Figure 6.** Begg’s funnel plot of publication bias in a selection of studies on the effects of artificial liver support systems on mortality. Each point represents a separate study for the indicated correlation. Log[RR], natural logarithm of relative risk (RR). Horizontal line, mean magnitude of the effect.

**Table I.** Characteristics of included studies in this meta-analysis.

First author	Year	Country	n		Subtype of HF	Etiology	Interventions	CONSORT score
			Treatment	Control				
Redeker *et al* (20)	1973	USA	8	20	AHF	Viral hepatitis	Transfusion (artificial)^a^	13
O’Grady *et al* (21)	1988	UK	29	33	AHF	Multi-etiology	Hemoperfusion (artificial)^a^	16
Davenport *et al* (22)	1993	UK	12	18	AHF	Multi-etiology	Hemofiltration (artificial)^a^	16
Hughes *et al* (23)	1994	UK	5	5	AHF	Drug induced liver disease/viral hepatitis	BioLogic-DT (artificial)^acd^	17
Ellis *et al* (24)	1996	UK	12	12	AHF	Multi-etiology	ELAD (bioartificial)^acd^	14
Mazariegos *et al* (25)	1997	USA	5	5	AHF	NR	BioLogic-DT (artificial)^a–c^	16
Kramer *et al* (26)	1998	Austria	10	10	AOCHF	Multi-etiology	BioLogic-DT (artificial)^a–d^	17
Wilkinson *et al* (27)	1998	USA	6	5	AHF	Multi-etiology	BioLogic-DT (artificial)^a–c^	17
Ellis *et al* (28)	1999	UK	5	5	AOCHF	Alcoholic liver disease	BioLogic-DT (artificial)^abd^	11
He *et al*-a (29)	2000	China	37	33	AHF	Viral hepatitis	Hemoperfusion/hemofiltration (artificial)^abd^	11
He *et al*-b (29)	2000	China	27	27	AOCHF	Viral hepatitis	Hemoperfusion/hemofiltration (artificial)^ad^	11
Mitzner *et al* (30)	2000	Germany	8	5	AOCHF	Multi-etiology	MARS (artificial)^ade^	16
Stevens *et al* (31)	2001	USA/Europe	73	74	AHF	Multi-etiology	HepatAssist (bioartificial)^acd^	12
Heemann *et al* (32)	2002	Germany	12	11	AOCHF	Multi-etiology	MARS (artificial)^acd^	17
Demetriou *et al* (33)	2004	Denmark	73	74	AHF	Multi-etiology	HepatAssist (bioartificial)^a^	18
El Banayosy *et al* (34)	2004	Germany	14	13	AHF	Cardiogenic shock	MARS (artificial)^ade^	11
Sen *et al* (35)	2004	UK	9	9	AOCHF	Alcoholic liver disease	MARS (artificial)^acd^	15
Laleman *et al* (36)	2006	Belgium	12	6	AOCHF	Alcoholic liver disease	MARS/Prometheus (artificial)^e^	13
Hassanein *et al* (37)	2007	Germany	39	31	AOCHF	Liver cirrhosis	MARS (artificial)^acd^	20
Kribben *et al* (38)	2012	Europe	77	68	AOCHF	Multi-etiology	Prometheus (artificial) ^ade^	21

a mortality,

b bridging to transplantation,

c hepatic encephalopathy,

d bleeding,

e total bilirubin (mg/dl). NR, not reported; HF, hepatic failure; AHF, acute hepatic failure; AOCHF, acute-on-chronic hepatic failure; MARS, molecular adsorbent recirculation system; ELAD, extracorporeal liver assist device; CONSORT, Consolidated Standards of Reporting Trials.

**Table II.** Univariate and multivariate meta-regression analyses of potential sources of heterogeneity.

Heterogeneity factor	Coefficient	SE	z	P-value	95% CI	
					UL	LL
Publication year						
Univariate	−0.005	0.015	−0.34	0.736	−0.034	0.024
Multivariate	0.032	0.063	0.51	0.613	−0.092	0.155
Country						
Univariate	0.077	0.073	1.05	0.293	−0.066	0.220
Multivariate	−0.059	0.256	−0.23	0.817	−0.562	0.443
Subtype of hepatic failure						
Univariate	−0.019	0.036	−0.52	0.603	−0.088	0.051
Multivariate	−0.024	0.065	−0.37	0.713	−0.150	0.103
Etiology						
Univariate	0.010	0.036	0.28	0.777	−0.059	0.080
Multivariate	−0.040	0.105	−0.38	0.704	−0.246	0.166
Interventions						
Univariate	−0.004	0.030	−0.13	0.893	−0.063	0.054
Multivariate	0.004	0.078	0.05	0.957	−0.148	0.156
CONSORT score						
Univariate	−0.044	0.033	−1.34	0.179	−0.108	0.020
Multivariate	−0.112	0.139	−0.81	0.419	−0.384	0.160

SE, standard error; 95% CI, 95% confidence interval; UL, upper limit; LL, lower limit; CONSORT, Consolidated Standards of Reporting Trials.
